# Jawbone microenvironment promotes periodontium regeneration by regulating the function of periodontal ligament stem cells

**DOI:** 10.1038/srep40088

**Published:** 2017-01-05

**Authors:** Bin Zhu, Wenjia Liu, Yihan Liu, Xicong Zhao, Hao Zhang, Zhuojing Luo, Yan Jin

**Affiliations:** 1 State Key Laboratory of Military Stomatology, Centre for Tissue Engineering, School of Stomatology, Fourth Military Medical University, Xi’an, Shaanxi, People’s Republic of China; 2 Department of Orthopedics Surgery, Xijing Hospital, Fourth Military Medical University, Xi’an, Shaanxi, People’s Republic of China; 3 Department of Stomatology, PLA Xizang Military Region General Hospital, Lhasa, Tibet, People’s Republic of China; 4 Department of Stomatology, PLA 301th Hospital, Beijing, People’s Republic of China

## Abstract

During tooth development, the jawbone interacts with dental germ and provides the development microenvironment. Jawbone-derived mesenchymal stem cells (JBMSCs) maintain this microenvironment for root and periodontium development. However, the effect of the jawbone microenvironment on periodontium tissue regeneration is largely elusive. Our previous study showed that cell aggregates (CAs) of bone marrow mesenchymal stem cells promoted periodontium regeneration on the treated dentin scaffold. Here, we found that JBMSCs enhanced not only the osteogenic differentiation of periodontal ligament stem cells (PDLSCs) but also their adhesion to titanium (Ti) material surface. Importantly, the compound CAs of PDLSCs and JBMSCs regenerated periodontal ligament-like fibers and mineralized matrix on the Ti scaffold surface, both in nude mice ectopic and minipig orthotopic transplantations. Our data revealed that an effective regenerative microenvironment, reconstructed by JBMSCs, promoted periodontium regeneration by regulating PDLSCs function on the Ti material.

During tooth development, root and periodontium formation is regulated by the development microenvironment^1^. This development microenvironment mainly consists of a biogenic signaling molecule from the interaction between ecto-mesenchyma and epithelium^2^,^3^. Jawbone derived from ecto-mesenchyma is critical for root development, especially periodontium tissue. It has been shown that tooth root may not completely develop in the absence of the jawbone microenvironment *in vivo* and vice versa^4^. Tissue regeneration is believed to occur due to the development of tissue substitutes that can mimic the structure and function of their natural analogues within the body^5^. Therefore, we hypothesize that the jawbone microenvironment promotes periodontium regeneration.

Mesenchymal stem cells (MSCs) participate in jawbone metabolism and maintain local microenvironment homeostasis. It has been reported that jawbone-derived MSCs (JBMSCs) had the ability of self-renewal and multi-lineage differentiation^6^. When jawbone homeostasis is broken, MSCs may be activated to differentiate into osteoblasts and secrete dozens of biomolecules, such as signal molecules, transcription factors, growth factors and extracellular matrix (ECM), to repair the structure and function of the jawbone^6^,^7^,^8^.

Periodontium tissue is necessary for tooth root regeneration, which can buffer the occlusal force and prevent progressive bone adsorption^9^. However, the periodontium, a complex composed of periodontal ligament (PDL), cementum, alveolar bone and gingiva, is difficult to regenerate integrally. Periodontal ligament stem cells (PDLSCs) and iliac bone-derived MSCs (IBMSCs) were reported to participate in periodontium tissue regeneration^10^,^11^,^12^,^13^, and their interaction also facilitated this process^14^. Our previous study proved that compound cell aggregates (CAs) of PDLSCs and bone marrow MSCs promoted periodontium regeneration with regenerative microenvironment reconstruction^15^. The favorable regenerative microenvironment was considered to induce seed/host cells self-assembly migration, tissue-affinitive differentiation, long-acting proliferation, and directed regulation by cytokines, which were helpful to complex tissue regeneration^16^,^17^,^18^.

In this study, to confirm the effect of the jawbone microenvironment on periodontium regeneration, we used inactive metal, titanium (Ti), as scaffold. We found that JBMSCs promoted osteogenic differentiation, adhesive rate and bio-function of PDLSCs on Ti samples. In addition, more mineralized matrix deposition and well-arranged PDL-like fibers were regenerated by compound CAs of JBMSCs and PDLSCs coated on Ti surface, both in nude mice ectopic and minipig orthotopic transplantations. In addition, higher successful rate of periodontium regeneration of compound CAs of jawbone- derived JBMSCs/and PDLSCs was shown in the minipig orthotopic transplantation. Therefore, we revealed that the CAs of JBMSCs provided a powerful regenerative microenvironment for periodontium regeneration via regulating the function of PDLSCs.

## Results

### Colony-forming ability, multilineage differentiation potentials, and surface markers of the PDLSCs, JBMSCs and IBMSCs

To identify the self-renewal potential of PDLSCs, JBMSCs and IBMSCs, the ability of colony-forming unit fibroblast (CFU-F) was determined (Figure S1A). The cells assumed a spindle-shape and single colonies formed 10 days after being plated at a low density of 10^3^ cells/well. With adipogenic induction, three MSCs can accumulate lipid droplets within the cytoplasm, as was confirmed by Oil Red O staining (Figure S1B). In addition, with osteogenic induction, three MSCs can form mineralized ECM, as was shown by staining with Alizarin Red (Kermel, Colmar, France) staining (Figure S1C). The PDLSCs, JBMSCs and IBMSCs positively expressed MSC-associated markers, including CD29, CD90 and CD105. PDLSCs expressed Stro-1 positively, and JBMSCs and IBMSCs expressed CD146 positively. Three MSCs all were negative for hematopoietic lineage markers, including CD34 and CD45, and platelet endothelial cell makers CD31 (Figure S2A,B and C).

### The initial adhesion and morphology of the PDLSCs on Ti indirectly co-cultured with JBMSCs/IBMSCs

PDLSCs were seeded indirectly co-cultured with JBMSCs or IBMSCs on Ti as the experiment groups and without co-culture on Ti as the control.

At 2 hours, PDLSCs of three groups on the Ti showed ball-like and few sharp short protrusions by scanning electron microscopy (SEM) (S-4800; Hitachi Ltd., Tokyo, Japan) (Fig. 1A). At 24 hours, PDLSCs extended longer and exhibited more long protrusions (Fig. 1B).

To observe the initial adhesion of PDLSCs on Ti samples indirectly co-cultured with JBMSCs or IBMSCs, PDLSCs were fixed and stained by Hoechst-33342 (Sigma, USA) after seeded 0.5 and 2 hours. There was no significant difference in the adherent cell number among the three groups at 0.5 hours (Fig. 1C,D). However, the adherent cell number of PDLSCs, indirectly co-cultured with JBMSCs was greatest at 2 hours (P < 0.05), and the experiment groups were both significantly greater than control (P < 0.05) (Fig. 1C,D).

### The cell cycle assay and proliferation of PDLSCs on Ti indirectly co-cultured with JBMSCs/IBMSCs

The effect of JBMSCs or IBMSCs on the cell cycle of PDLSCs on Ti was also observed, at 4 days of co-culture (Figure S2A). There was no obvious difference in the percentage of S + G2 phases between two experiment groups (43.34% and 45.92%) for PDLSCs indirectly co-cultured with IBMSCs and JBMSCs respectively. The control group (40.92%) was slightly lower than the experiment groups. PDLSCs were fixed and stained by EdU-Apollo567 staining for proliferation assay, at 4 days of co-culture. The results showed no obvious proliferation difference among control and two experiment groups (Figure S2B). The effect of JBMSCs or IBMSCs on the proliferation of PDLSCs on Ti was assayed by 3-(4, 5-dimethylthiazol-2yl)-2, 5-diphenyltetrazolium bromide (MTT) and the Cell-Light TM EdU-Apollo567 Imaging Kit (RiboBio, Guangzhou, China). The MTT results showed slightly higher proliferation of PDLSCs indirectly co-cultured with JBMSCs at day 3, 4 and 5 (P < 0.05). There were no significant differences at other time points (Figure S2C).

### The osteogenic differentiation of PDLSCs on Ti indirectly co-cultured with JBMSCs/IBMSCs

To investigate the effect of JBMSCs or IBMSCs on osteogenic differentiation of PDLSCs on Ti, three MSCs were seeded in indirect co-culture system as control and two experiment groups with osteogenic induction.

Alkaline (ALP) staining of PDLSCs in three groups increased from day 7 to day 14 (Fig. 2A). ALP activity of PDLSCs, indirectly co-cultured with JBMSCs, was highest after 7 and 14 days of osteogenic induction. And ALP activity of both experiment groups were higher than control after 14 days of osteogenic induction (Fig. 2C) (P < 0.05). After 28 days, Alizarin Red staining showed significant difference among three groups (Fig. 2A,B)(P < 0.05). The expression levels of osteoblast-related genes, including runt-related transcription factor 2 (Runx2), ALP, type I collagen (Col-I) and periostin were determined by the real-time quantitative reverse-transcription polymerase chain reaction (qRT-PCR) analysis after 7 and 14 days of osteogenic induction (Fig. 2D,E). The gene expression analysis showed the same following result: PDLSCs indirectly co-cultured with JBMSCs, expressed higher levels of Runx2, ALP and Col-I at the 7 days of osteogenic induction (P < 0.05) (Fig. 2D). The level of ALP and Col-I decreased but was still significantly different from the two experiment groups at the 14days of culture. The periostin level increased and showed obvious difference between two experiment groups (P < 0.05). Further, these osteogenic gene expressions of both experiment groups were higher than the control (P < 0.05) (Fig. 2E).

### The bio-functional markers of CAs of PDLSC with JBMSCs/IBMSCs

The hematoxylin and eosin (H&E) staining showed that both CAs of PDLSCs with JBMSCs/IBMSCs were dense and contained plenty of cells, which could ensure the collagen secretion, and these compound CAs had at least 3 to 5 layers of cells (Fig. 3A).

Immunohistochemical analyses showed that compared with control, both compound CAs (Fig. 3B) positively expressed ALP (Fig. 3C), early markers for osteogenic differentiation; periostin, a special marker of PDL (Fig. 3E); integrinβ1 and fibronectin (Fig. 3D,F), markers related to the bio-function of CA; and runt-related transcription factor 2 (Runx2), a transcription factor of Wnt signal pathway (Fig. 3G).

### Morphology of compound CAs of PDLSCs with JBMSCs/IBMSCs grown on scaffolds *in vitro*

SEM analysis of ceramic bovine bone (CBB), the outer scaffold of transplant in nude mice, showed a porous structure (Fig. 4A). Differently, the surface of Ti-implant showed a micro-pore facial structure (Fig. 4B). The SEM images showed that two compound CAs contained a large number of cells and ECM. The compound CAs integrally adhered to the scaffolds and extended excessively on the surface of Ti and CBB (Fig. 4C–F).

### Periodontium-like tissue regeneration of compound CAs of PDLSCs with JBMSCs/IBMSCs on Ti in nude mice

Eight weeks after transplantation, 17/20 experiment specimens were harvested in the experiment groups and examined by Verhoeff-van Gieson (VVG) and Masson trichrome staining. In the CAs of PDLSCs with JBMSCs, a large number of well-arranged and dense collagen fiber (CF) bundles, which were more closely resembled the physiological structure of natural PDL tissue, formed between the surfaces of Ti-implant and CBB. Moreover, there were abundant blood vessels among the PDL-like fibers. In contrast, the CAs of PDLSCs with IBMSCs formed loose and disorderly arranged fibers between the Ti-implant and CBB, indicating poor periodontium tissue regeneration. There was seldom CF between surfaces of Ti and CBB in the control group (Fig. 5A,B), which suggested that no periodontium tissue regeneration formed.

Furthermore, Micro-CT 3D reconstruction images showed that newly formed mineralized matrix covered 56.5% of the Ti-implant surface of CAs of PDLSCs with JBMSCs on average, which was significantly higher than the CAs of PDLSCs with IBMSCs (42.3% on average) (P < 0.05). In addition, only 6.8% of newly formed mineralized matrix of the control group, without CA covered (Fig. 5C,D).

Additionally, the success rate of Ti with CAs of PDLSCs with JBMSCs or IBMSCs on periodontium regeneration in nude mice ectopic transplantation was calculated. However, there was no obvious difference (Table 1).

### Periodontium-like tissue regeneration of CAs of pig PDLSCs with JBMSCs/IBMSCs on Ti in minipigs

The Ti-implants, coated with compound CAs of pig PDLSCs with JBMSCs/IBMSCs were implanted into the minipig alveolar bone (Fig. 6A). Four experiment complexes grew well and solid, and showed a well-keratinized oral epithelium. All 20 Ti-implants were harvested after 12 weeks orthotopic transplantation in experiment groups. VVG and Masson trichrome staining showed that the autologous CAs of pig PDLSCs with JBMSCs regenerated a dozen of, well-arranged and dense CF on the Ti surface. These PDL-like fibers could integrate Ti-implant with alveolar bone closely together. However, there was a large amount of parallel collagen fibers around the Ti-implant in the autologous compound CAs of PDLSCs with IBMSCs. And there was osseointegration of the surfaces of the Ti and jawbone (Fig. 6B,C).

Additionally, Micro-CT 3D reconstruction results showed that newly formed mineralized matrix of CAs, of pig PDLSCs with JBMSCs, was greater than that of CAs of pig PDLSCs with IBMSCs (P < 0.05). However, the control group showed a much higher newly formed mineralized matrix contact rate (76.3%) than the experiment groups (Fig. 6D,E).

Furthermore, the regenerative success rate of CAs of PDLSCs with JBMSCs (8/10) on Ti-implant orthotopic transplantation was significantly higher than CAs of PDLSCs with IBMSCs (6/10) (P < 0.05) (Table 1). In addition, 9/10 of Ti without CAs got osseointegration between the surfaces of Ti-implant and alveolar bone.

## Discussion

The periodontium tissue consists of the periodontal ligament, alveolar bone, cementum and gingiva, and is difficult to regenerate as a complex tissue. With tissue-specific MSCs and tissue engineering technology, cell sheet of PDLSCs, bone marrow MSCs and dental follicle cells were used for periodontium regeneration and much achievement has been obtained^11^,^13^,^19^,^20^. However, the stability and function of these periodontium regeneration remained doubtful^21^. In a previous study, we successfully regenerated periodontium-like tissue on the osteogenic-induction scaffold CBB and treated dentin matrix^15^. In this study, we found JBMSCs enhanced the initial adhesion and osteogenic differentiation of PDLSCs on Ti. And compound CAs of JBMSCs/PDLSCs regenerated periodontium-like tissue on the inactive metal, Ti surface, both in nude mice ectopic and minipig orthotopic transplantations.

The initial adhesion of anchorage-dependent cells is a pivotal process for their subsequent function^22^. In this study, there was no difference on adhesive cell number among three groups at first 0.5 hours. And the adhesive cell number was elevated at 2 hours. The initial adhesion would affect differentiation and this was closely relative with tissue regeneration. And the growth factors and material surface treatment were well-recognized approaches to enhance the cell adhesion^23^. It was demonstrated that MSCs could induce cell adhesion of different cell types by both cell-cell contact and non-contact ways^24^,^25^,^26^,^27^. Here PDLSCs adhesion on Ti was promoted by JBMSCs via non-contact way. Some cytokines were believed to contribute to this process. The specific mechanism will be investigated. The shape of PDLSCs showed no obvious difference among three groups. At early stage, PDLSCs showed ball-like shape on Ti, and well-spread at 24 hours. And well-spread shape was thought to be closely relative with osteogenic differentiation^28^,^29^.

Mineralized matrix deposition on scaffold was the basis of cementum-PDL complex regeneration^30^. Therefore, the promotion of osteogenic or cementogenic differentiation of PDLSCs played an important role. In this study Alizarin Red staining, ALP staining and ALP activity assay showed osteogensis of PDLSCs was enhanced by JBMSCs via non-contact way. The qRT-PCR showed the gene expression level of ALP was still elevated at 7 and 14 days of indirect co-culture. However ALP was an early marker for osteogenic differentiation. The full understanding of this phenomenon was not obtained. And we guessed this would be relative with cytokines continuously secreted by JBMSCs. Previous studies showed MSCs would promote the osteogenic differentiation of various kinds of cells by both direct and indirect co-culture^31^,^32^,^33^. And some researchers have focused on the osteogenic induction potential of odontogenic MSCs, which prepared for periodontium tissue regeneration^34^. Some underlying cytokines were thought to be secreted to facilitate this process, which will be discussed in further study.

In this study, the cell cycle analysis and EdU-Apollo567 staining results showed the high level of proliferative activity in three groups, indicating good biocompatibility of Ti and favorable cell viability of PDLSCs. The MTT result showed significant difference between two experiment groups, which indicated promotion of cell viability was brought by compound CAs of PDLSCs with JBMSCs. However, no obvious difference was observed in the cell cycle analysis and EdU-Apollo567 staining. This may be explained by the reciprocal relationship between cell proliferation and differentiation^35^.

It was demonstrated that, compared with odontogenic cells, odontogenic CAs expressed more bio-functional markers, including ALP, bone sialoprotein, osteopontin, Runx2, type III collagen and periostin, which would facilitate the periodontium regeneration^36^. Here the compound CAs composed of plenty of MSCs and ECM. The seed cells and ECM provided CAs with a regeneration origin and great mechanical and biological properties, respectively. Fibronectin and integrinβ1 could promote migration and proliferation of MSCs in CAs^37^,^38^,^39^. Periostin, an adhesion molecule for preosteoblats, represented an important marker for fibroblastic cells in the PDL and osteoblasts on the alveolar bone surface^40^. ALP was major molecule of osteogenic differentiation which was involved in Wnt signal pathway^41^. These biological properties of compound CAs facilitated periodontium regeneration.

In the construction of compound CAs, PDLSCs, JBMSCs and IBMSCs were cultured into mono type CAs first, and then they were compounded layer by layer. The different types of cells could contact directly on the surfaces of the mono type CAs. This formation was quite different from the traditional cell-cell contacting style between two different cell types. Even so we cannot exclude the cell-cell contact function, which would contribute to periodontium regeneration of the compound CAs. Previous studies showed that direct co-culture with MSCs would promote osteogensis^31^,^42^. And the mixture CAs of different cell types will be an appropriate model for cell-cell contact study.

Most of periodontium regeneration experiments were based on osteogenic induction material, such as treated dentin matrix, CBB and β-hydroxylapatite actually^11^,^13^,^14^,^15^,^30^,^43^. These materials induced periodontium regeneration of PDLSCs strongly. Ti possessed great biocompatibility and osteogenic induction^44^, but inactive odontogenic induction. In addition, periodontium regeneration was seldom reported on the Ti, and the researches focused on the osteogenic coating and modified surface treatment instead^45^,^46^,^47^. Our previous study showed PDLSCs with JBMSCs had an advantage in periodontium regeneration. Therefore, to verify the microenvironment provided by JBMSCs, Ti was chosen as the scaffold. It was reported that the whole tooth grew up with physiological structure and function when dental germ tissue was kibbled into epithelium and mesenchyme, then mixed and implanted into the alveolar cavity of mice^48^,^49^,^50^. It was suggested that the interaction between epithelium and mesenchyme, under a favorable microenvironment, would recover from irregular and disorderly tissue arrangement. Our data showed JBMSCs promoted adhesion and osteogenic differentiation of PDLSCs on the Ti in the indirect co-culture system, which suggested that JBMSCs reconstructed the regenerative microenvironment via the non-contacting approach to regulate the function of PDLSCs. Moreover, a large amount of well-arranged and dense CF bundles and mineralized matrix deposition were regenerated by CAs of PDLSCs with JBMSCs in both ectopic and orthotopic implantations. Additionally, a higher periodontium regeneration success rate on was shown. The results demonstrated CAs of jawbone-derived MSCs/PDLSCs were an optimal choice for periodontium regeneration. However, the specific mechanism of microenvironment reconstructed by JBMSCs is still unclear. This issue will be focused on in our future research.

## Conclusion

The adhesion and osteogenic differentiation of PDLSCs on the Ti were enhanced by JBMSCs via non-contacting approach. The periodontium tissue regeneration by compound CAs of PDLSCs with JBMSCs on the Ti was observed in the ectopic and orthotopic implantation models. This study demonstrated that jawbone microenvironment promoted periodontium regeneration and provided a strategy for periodontium regeneration on the inactive material bio-tooth.

## Materials and Methods

### Ethics Statement

Written informed consent was provided by all participants, and ethical approval had been obtained from the Ethics Committee of the School of Stomatology, the Fourth Military Medical University, Xi’an, China. All the methods in the study were carried out in accordance with the approved guidelines.

All animal procedures were performed in accordance with the approved guidelines of the Animal Care Committee of the Fourth Military Medical University, Xi’an, China.

### Scaffold materials preparation

Pure Ti plates (10 × 10 × 1 mm^3^) and Ti rods (Φ 2 × 4 mm^3^) (99.9%) (Zhong Bang biomaterials technology company, Xi’an, People’s Republic of China) were used in our study. The roughness surface of the Ti-implant was obtained by a sandblasting large-grit acid-etching (SLA) technique^51^. The samples were sterilized with cobalt-60 before the cell plating and animal studies.

The CBB (Research and Development Center for Tissue Engineering, Fourth Military Medical University, Xi’an, China) tubes were produced from fresh bovine rib bones, which were subsequently cut into blocks, washed in normal saline and soaked in H_2_O_2_ to remove proteins. Next, the blocks were remodeled into hollow tubes through a high-speed drill (height of 7.0 mm, internal diameter of 3.0 mm, outside diameter of 8.0 mm). These deproteinized hollow tubes were washed with running water, heated at 900 °C for 1 hour, and sterilized in a high temperature and pressure environment before using^15^.

### Cell culture

All procedures of cell culture and identification, of both humans and minipigs, were the same as the previous description^7^,^12^,^52^.

Healthy human tooth samples were collected from 10 donors, aged from 15 to 24 years, undergoing routine premolar or third molar extractions for orthodontic reasons. Iliac bone marrow samples were collected from 10 donors, aged from 18–30 years, undergoing alveolar bone cleft repair by auto-ilium transplantation. Human jawbone samples were obtained from the patients who had undergone orthognathic surgery (10 donors aged 18–28 years). In addition, five, 2-year-old minipigs were used for the pig relative cell culture.

In brief, PDL tissues were gently separated from the surface of the mid-third of the root, and subsequently digested with 3 mg/ml of collagenase type I (Sigma, St. Louis, MO, USA) for 60 min at 37 °C and then cultured in α-minimum essential medium (α-MEM, Gibco BRL, Gaithersburg, MD, USA) supplemented with 15% fetal bovine serum (FBS; FBS, Gibco, BRL), 0.292 mg/ml glutamine (Invitrogen, Carlsbad, CA, USA), 100 U/ml penicillin, and 100 mg/ml streptomycin (Invitrogen, Fredick, USA) in 6-well culture dishes (Costar, USA) at 37 °C in a humidified atmosphere of 5% CO_2_ and 95% air. After 2 weeks in culture, cells from PDL became subconfluent. To obtain homogeneous populations of PDLSCs, single cell-derived colony cultures were obtained using the limiting dilution technique.

A total of 1 mL iliac bone marrow aspirates was seeded into a 10 cm culture dish, and 20 mL α-MEM (Gibco BRL, Gaithersburg, MD) was added, supplemented with 15% FBS (Gibco BRL, Gaithersburg, MD) and then incubated in 5% CO_2_, 37 °C.

Jawbone debris was rinsed 3 times with α-MEM (Gibco BRL, Gaithersburg, MD), containing 100 U/mL of penicillin and 100 mg/mL of streptomycin (Invitrogen, Frederick, MD, USA). The debris was cut into almost 1 × 1 mm^2^ pieces and passed through a 70 μm strainer to obtain single cell suspensions. Both the cell suspensions and jawbone pieces were seeded into a 10 cm diameter culture dish and cultured as IBMSCs. Multiple colony-derived human and pig MSCs at 2–4 passages were used in our experiments. All the experiments in this study were replicated at least 3 times.

### Identification of PDLSCs, JBMSCs and IBMSCs

#### Colony-forming efficiency test

To assess the ability to produce colony-forming units, single-cell suspensions (1 × 10^3^ cells) were seeded in 10 cm diameter culture dishes. After 14 days of culture, three MSCs were fixed in 4% paraformaldehyde and stained with 0.1% toluidine blue for 30 min. After being washed with phosphate-buffered solution (PBS), images were taken by stereoscopic microscope (Nikon, Japan).

#### Flow cytometry (FCM) analysis

To characterize the immunophenotype of *in vitro*-expanded PDLSCs, JBMSCs and IBMSCs, FCM analysis was performed to assay the expression of MSC-associated surface markers at early passages (P3). Briefly, the adherent cells were washed twice with PBS and liberated by 2 mL of 0.05% trypsin (Sigma-Aldrich Corp). Then, the single-cell suspension was washed twice and resuspended in PBS containing 3% FBS. For the identification of the MSC phenotype, approximately 5 × 10^5^ PDLSCs, JBMSCs or IBMSCs/200 μL of PBS in each EP tube were incubated with phycoerythrin or fluorescein isothiocyanate-conjugated monoclonal antibodies for human CD29, CD31, CD90, CD146 (Bioscience, San Diego, CA, USA), CD34, CD45 and CD105 (BioLegend, San Diego, CA, USA) for 1 hour at 4 °C in the dark. Additionally, STRO-1 (BioLegend, San Diego, CA, USA) was assayed for PDLSCs alone. The cells without any antibodies were used as negative control. Then, the cells were washed twice with 1 mL PBS. Finally, the labeled cells were analyzed by FCM (Becton Coulter Inc., Brea, CA, USA).

#### Adipogenic differentiation

To induce adipogenic differentiation, at 70% confluence three MSCs were respectively cultured in α-MEM supplemented with 10% FBS, 2 μm insulin, 0.5 M isobutylmethylxanthine and 10 nM dexamethasone for 21 days. Then the cells were washed twice with PBS and fixed in 4% paraformaldehyde for 60 min. Oil red O (Sigma-Aldrich Corp) staining was performed, and then lipid droplets were identified microscopically.

#### Osteogenic differentiation

To induce osteogenic differentiation, after reaching 70% confluence, three MSCs were respectively cultured in α-MEM supplemented with 10% FBS, 100 nM dexamethasone, 50 μg/mlascorbic acid and 5 mM β-glycerophosphate for 28 days. The medium was changed every 3 days. Calcium accumulation was detected by 2% Alizarin Red (Kermel, Colmar, France)staining. After washed with distilled water three times, stained calcium nodules were identified microscopically.

### Construction of indirect co-culture system of PDLSCs, JBMSCs and IBMSCs on Ti

First, the sterilized Ti plate was put in the well of a 24-well plate. Then, PDLSCs were seeded on the Ti plate surface at 10^4^ cells/well. Then, the Transwell filters (6.5 mm internal diameter, 0.4 μm pore size) (Corning, Incorporation, NY, USA) were hung in the well of a 24-well plate and seeded with JBMSCs or IBMSCs in the Transwell chamber at 10^4^ cells/well (Figure S3D). The indirect co-culture system was cultured with α-MEM with 10% FBS.

### Adhesion and morphology of PDLSCs indirectly co-cultured with JBMSCs/IBMSCs on Ti

After three MSCs were seeded in the indirect co-culture system for 0.5 and 2 hours, as described above, the Ti plates were washed with PBS three times, fixed in 4% glutaraldehyde for 4 hours and then stained with Hoechst-33342. The cell numbers on each plate were counted in three random 5+ fields under an epifluorescence microscope (Leica Microsystems, Wetzlar, Germany) after seeded 0.5 and 2 hours.

After seeded in the indirect co-culture system on Ti 2 and 24 hours, PDLSCs were dehydrated in a graded ethanol series, freeze-dried and sputter coated with gold, prior to observation by SEM (S-4800; Hitachi Ltd., Tokyo, Japan).

### Cell proliferation of PDLSCs indirectly co-cultured with JBMSCs/IBMSCs on Ti

The MTT assay was used to test the effect of JBMSCs or IBMSCs on PDLSCs’ proliferation. Briefly, three MSCs were seeded in the indirect co-culture system and cultured by 1500 μL α-MEM with 10% FBS (covered the bottom of Transwell filters). On days 1 to 7, 150 μL of MTT solution (Sigma-Aldrich, 5 mg/mL) was added to each well and incubated at 37 °C for 4 hours. Then, the medium was discarded, and formazan salts were dissolved in 200 μL of dimethyl sulfoxide (DMSO, Sigma-Aldrich). The absorbance in individual wells was read at 540 nm by a microplate reader (ELx800, BioTek Instruments Inc., USA) and expressed as optical density with Soft Max Pro software.

The incorporation of 5-ethynyl-2′-deoxyuridine (EdU), a thymidine analog, can label cells undergoing DNA replication. The Cell-Light^TM^ EdU-Apollo567 Imaging Kit (RiboBio, Guangzhou, China) was used to confirm the effect of JBMSCs or IBMSCs on PDLSCs’ proliferation. Three MSCs were seeded in the indirect co-culture system for 4 days. Then, 1500 μL α-MEM with EdU (50 μM) was added to each well for 2 h. The EdU medium mixture was discarded, and 4% paraformaldehyde was added for 30 min at room temperature to fix the cells. The cells were washed with glycine (2 mg/ml) for 5 min in a decolorization shaker, 0.5% Trion X-100 was added for 10 min, and the cells were washed twice with PBS. Next, 100 μL EdU-Apollo567 stain reaction buffer was added to each well for 30 min while shielding from light. The cells were washed three times with 0.5% Triton X-100 for 30 min at room temperature; 200 μL PBS was then added. FCM analysis was performed to detect and assay fluorescence staining cells at 550 nm.

### Cell cycle analysis of PDLSCs indirectly co-cultured with JBMSCs/IBMSCs on Ti

Three MSCs were respectively seeded in the indirect co-culture system. At 4 days of co-culture, the PDLSCs on six plates for each group were trypsinized and pooled for cell cycle analysis. After washing with PBS, the PDLSCs were resuspended in 1 mL of PBS with repeated vibration to get a suspension. The cells in the suspension were fixed with ice-cold dehydrated ethanol overnight at 4 °C. The fixed cells were washed twice with PBS and stained with 100 mg/mL propidium iodide (PI) (Sigma-Aldrich Corp) at 4 °C for 30 minutes. The PI-elicited fuorescence of individual cells was measured using FCM. At least 5 × 10^5^ cells were analyzed for each sample. The amounts of cells residing in the G0/G1 phase, S phase, and G2 phase were determined.

### Osteogenic differentiation of PDLSCs indirectly co-cultured with JBMSCs/IBMSCs on Ti

To induce osteogenic differentiation in indirect co-culture system, after cells reached 80% confluence, the culture medium was changed to the α-MEM supplemented with 10% FBS, 100 nM dexamethasone, 50 μg/ml ascorbic acid and 5 mM β-glycerophosphatefor 28 days. The medium was changed every three days. Calcium accumulation was detected by 2% Alizarin Red staining and dissolved in 1 mL of sodium dodecyl sulfate solution. The light absorption of sodium dodecyl sulfate solution with Alizarin Red was read at 570 nm with a microplate reader (Bio-TEK Instruments, Winooski, VT, USA). The quantitative analysis of Alizarin Red staining was normalized by initial seeding cell number. Ti with PDLSCs were washed twice in PBS after fixation in 4% paraformaldehyde for 20 min. ALP staining was determined with the BCIP/NBT Alkaline Phosphatase Color Development Kit (Beyotime Co., Shanghai, China). In addition, ALP activity was determined by ALP activity detection kit (Jiancheng Bioengineering Institute, Nanjing, People’s Republic of China), according to the manufacturer’s suggested protocols. ALP activity was normalized by protein concentration.

### The gene expression of PLDSCs indirectly co-cultured with JBMSCs/IBMSCs on Ti

The expression of genes, including Runx2, ALP, periostin and type I collagen, was determined by qRT-PCR analysis^52^. PDLSCs, indirectly co-cultured with JBMSCs or IBMSCs on Ti, were cultured in osteogenic medium and harvested at 7 and 14 days at density of 10^5^/well. And PDLSCs were culture on theTi without co-culture in osteogenic medium as control. All PDLSCs were harvested using TRIzol (Gibco®; Life Technologies Corp, Carlsbad, CA, USA) to extract the RNA. An equivalent amount of RNA from each sample was reverse transcribed into complementary DNA (cDNA) using a Superscript II first-strand cDNA synthesis kit (Invitrogen®; Life Technologies Corp). The qRT-PCR analysis on the genes above was performed on the Applied Biosystems 7500 using the QuantiTect® Sybr® Green Kit (Qiagen, Venlo, the Netherlands). The primers for the target genes were listed in Table 2. The expression levels of the target genes were normalized to that of the housekeeping gene β-actin.

### Construction of the compound CAs of PDLSCs with JBMSCs/IBMSCs

Multiple colony-derived three MSCs from both humans and minipig at passage 3 were seeded at approximately 1 × 10^5^/mL into 12-cell plates, respectively. After reaching 90% confluence, the medium was changed into CAs induction medium, containing 10% FBS and ascorbate (50 μg/ml). Finally, the mono cell type CAs formed in 2 weeks and easily detached from the culture plates with a cell scraper. The construction of JBMSCs or IBMSCs CAs were similar to the PDLSCs CAs. The compound CAs contained 2 layers of PDLSCs CAs and 1 layer of JBMSCs or IBMSCs CAs outside. The compound CAs were put into double collagen pallets, which constituted a collagen-CAs-collagen ‘sandwich,’ and then cultured with osteogenic induction media for 1 week.

### H&E and immunohistochemical staining of the compound CAs

The collagen-CAs-collagen ‘sandwiches’ were fixed in 4% paraformaldehyde for 24 hours, paraffin-embedded, longitudinally sectioned and stained with H&E. Other sections were incubated with primary antibodies follows anti-ALP (1:200, Abcam, British), anti-periostin (1:200, Santa, USA), anti-fibronectin (1:200, Abcam, British), anti-Runx2 (1:200, Abcam, British) and anti-integrin β (1:200, Abcam, British). PBS was used for the negative controls instead of the primary antibodies. Bio-tinylated secondary antibodies (1:1000) were purchased from Dako (Dako, USA). The staining sections were observed with a light microscope (Nikon, Japan).

### Observation of the compound CAs with scaffold Ti-implant/CBB via SEM

The inner-scaffold Ti-implant was coated by one layer of PDLSCs CAs. Then, this complex was coated by another layer of PDLSCs CAs. Next, this complex was coated by one layer of JBMSCs or IBMSCs CAs outside. Finally, the Ti implant with compound CAs was inserted into a CBB tube (Fig. 4G). The entire complex was cultured in osteogenic medium for 7 days and then fixed in 4% paraformaldehyde. The samples were anodized in an electrolyte containing 0.5 wt % hydrofluoric acid and 1 M phosphoric acid for 1 h. After that, the whole complex was observed by SEM.

### Nude mice ectopic transplantation

All the animal procedures complied with the guidelines provided by the Animal Care Committee of the Fourth Military Medical University. The complex implants, including inner scaffold Ti-implant, compound CAs and outer scaffold CBB tube, were subcutaneously transplanted into the dorsal surface of ten 8-week-old nude mice (BALB/c-nu; FMMU Medical Laboratory Animal Center, Xi’an, China). Control implants without compound CAs were subcutaneously transplanted into both sides of the dorsal surface of another five, 8-week-old nude mice. All nude mice were injected with 0.1 μg/g mebumalnatrium for anesthesia. The implants with compound two CAs of two experiment groups were transplanted into different sides of subcutaneous pockets separately. After eight weeks of the transplantation, all fifteen nude mice were euthanized, and all 30 implants were removed for analysis.

### Minipig orthotopic transplantation

Under local anesthesia, four canine teeth were extracted from each of five 2-year-old minipigs, 3 months before the present experiments. The PDLSCs, JBMSCs or IBMSCs were isolated and the compound pig CAs of PDLSCs with JBMSCs or IBMSCs were constructed, as previously described^15^. All five pigs were intramuscularly injected with 0.1 mg/kg medetomidine (Sigma) and 15 mg/kg ketamine (Sigma) for anesthetic premedication and then subjected to an intravenous injection of 2.5 mg/kg propofol (Sigma). An endotracheal tube was inserted. Following alveolar bone exposure, the implant site was prepared with a round bur (1.9 mm diameter) and custom-made drill (2.0 mm diameter) with mountable stop (4 mm). Ti-implants (2.0 mm × 4.0 mm), coated by autologous compound CAs of two experiment groups were implanted into fabricated molded wells (2.0 mm diameter) on the different sides of mandibula separately. Implant beds were prepared to avoid friction during implantation, and the implants were quite stable (Fig. 6A). The control Ti implants without autologous compound CAs were also implanted into both sides of the mandibula. All the implants of each minipig were harvested after 12 weeks.

### Micro-CT analysis for mineralized matrix deposition on Ti

The Ti-implants of three groups were harvested from nude mice and minipigs respectively, and then fixed with 4% paraformaldehyde for 2 days. Each sample was then scanned by micro-CT (Siemens, Germany) to examine the newly-formed mineralized matrix deposition on the Ti surface. Three-dimensional (3D) reconstructions of the samples were performed using COBRA (Siemens, Germany).

### Morphological and Histomorphometric evaluation of regenerated PDL-like tissue

The implants were fixed in a solution of 10% formaldehyde at room temperature for 7 days. Then, they were dehydrated in a graded ascending ethanol series (70–100%), infiltrated and embedded in methyl methacrylate (MMA). Serial sections (150 μm) along the horizontal axis were made using a high-speed precision microtome (LEICA SP1600, Germany). All the sections were ground and polished into 35 μm then stained with VVG and Masson trichrome staining.

Briefly, the sections were stained for 30 min in Verhoeff’s solution (4% alcoholic hematoxylin (20 ml), 10% aqueous ferric chloride (8 mL), 2 g Lugol’s iodine, 4 g potassium iodine, 100 mL distilled water (8 mL)). Then differentiated in 2% ferric chloride (Sigma-Aldrich) for 1 min, and washedin running tap water for 1 min. The sections were placed in 95% alcohol to remove iodine stain. Then washed in running tap water for 1 min. Counterstained in Van Gieson solution (1% aqueous solution of acid fuchsin (10 ml), saturated aqueous solution of picric acid (200 ml)) for 3 to 5 min. Dehydrated through serial solutions of graded alcohols, clear with xylene, dry, and coverslip.

Briefly, stained nuclei with celestin blue-hematoxlyin. Then differentiated with 1% acid alcohol and washed in running tap water for 1 min. Stainedthe section with solution A (acid fuchsin (0.5 g), glacial acetic acid (0.5 ml), distilled water (100 ml)) for 5 min and then rinsed in distilled water. Treated with solution B (phosphomolybdic acid (1.0 g), distilled water (100 ml)) for 5 min and then rinsed in distilled water. Stained the section with solution C (methyl blue (2.0 g), glacial acetic acid (2.5 ml), distilled water (100 ml)) for 3–5 min and treated with 1% acetic acid for 2 min. Dehydrated through serial solutions of graded alcohols, clear with xylene, dry, and coverslip.

A microscope (Leica Microsystems AG, Wetzlar, Germany) was used for histological evaluation, which was based on the morphological observation of three sections per implant.

### Statistical analysis

All the statistical analyses were performed using ANOVA followed by Fisher’s protected least significant difference test and student’s t-test by SPSS version 15.0 software (SPSS, USA). All the values are expressed as mean ± SD. A P-value < 0.05 was considered to be statistically significant.

## Additional Information

**How to cite this article**: Zhu, B. *et al*. Jawbone microenvironment promotes periodontium regeneration by regulating the function of periodontal ligament stem cells. *Sci. Rep.* **7**, 40088; doi: 10.1038/srep40088 (2017).

**Publisher's note:** Springer Nature remains neutral with regard to jurisdictional claims in published maps and institutional affiliations.

## Supplementary Material

Supplementary Figures

## Figures and Tables

**Figure 1:** Initial adhesion and morphology of PDLSCs on Ti in indirect co-culture system. Morphology of PDLSCs and PDLSCs indirectly co-cultured with JBMSCs/IBMSCs after 2 hours (**A**) and 24 hours (**B**) by SEM. Adhesive number of PDLSCs in indirect co-culture system were measured by counting the Hoechst-stained cells under a fluorescence microscope after 0.5 and 2 hours (**C,D**). The data are shown as the mean ± SD; *P < 0.05, n = 3.

**Figure 2:** Osteogenic differentiation of PDLSCs on Ti in indirect co-culture system. ALP staining (**A**) and ALP activity (**C**) test were performed after 1 and 2 weeks of osteogenic induction, respectively. Alizarin Red staining (**A**) and quantitative analysis (**B**) were performed after 4 weeks of osteogenic induction. The expression levels of Runx2, ALP, Col-I and periostin investigated by qRT-PCR after PDLSCs indirectly co-cultured with JBMSCs/IBMSCs on Ti. The expression levels were normalized to β-actin with osteogenic induction for 1 (**D**) and 2 weeks (**E**). The data are shown as the mean ± SD; *P < 0.05, n = 3.

**Figure 3:** Immunohistochemical analyses of compound CAs. Both compound CAs positively expressed ALP, fibronectin, periostin, integrinβ1 and Runx2. ALP and Runx2 indicated the osteogenic differentiation capacity. Integrinβ1 and fibronectin were the markers of bio-functions. Periostin was a special marker of periodontal ligament.

**Figure 4:** Microscopic appearance of the scaffold materials and the adhesion of the compound CAs to the scaffolds. SEM images of CBB showed a porous structure, while Ti-implant showed a micro-pore facial structure (**A,B**). The attachment of compound CAs on the surface of CBB or Ti-implant was analyzed by SEM (**C–F**).

**Figure 5:** Periodontium tissue regeneration of compound CAs in nude mice ectopic transplantation. Periodontium regeneration of human compound CAs, and the control group was analyzed by VVG (**A**) and Masson trichrome (**B**) staining. Reconstructive images showed mineralized matrix deposition on Ti (**C**). The quantitative assay of reconstruction images showed the average difference of mineralized matrix on Ti was significant among three groups (P < 0.05) (**D**). The red arrows indicate blood vessel. The data are shown as the mean ± SD; *P < 0.05, n = 3.

**Figure 6:** Periodontium tissue regeneration of compound CAs in minipig orthotopic transplantation. The transplantation surgery on minipigs was shown (**A**). Periodontium regeneration of pig compound CAs was analyzed by VVG (**B**) and Masson trichrome (**C**) staining. Reconstructive images showed mineralized matrix position on the Ti (**D**). The quantitative assay of reconstruction images showed the average difference of mineralized matrix on Ti was significant among three groups (P < 0.05) (**D**). The red arrows indicate blood vessel. The data are shown as the mean ± SD; *P < 0.05, n = 3.

**Table 1:** Compound CAs coating Ti in nude mice ectopic transplantation and minipig orthotopic transplantation success rate.

Group	hJBMMSCs/hPDLSCs with Ti	hIBMMSCs/hPDLSCs with Ti	pJBMMSCs/hPDLSCs with Ti	pIBMMSCs/hPDLSCs with Ti
Implant	10	10	10	10
Die	1	1	0	0
Lost	0	1	0	0
Harvest	9	8	10	10
Regeneration	8	7	8	6
Success rate	88.9%	87.5%	80.0%	60.0%

**Table 2:** Primer Sequences.

Gene	Forward	Reverse
RUNX2	5′-CCCGTGGCCTTCAAGGT-3′	5′-CGTTACCCGCCATGACAGTA-3′
Periostin	5′-GCTGCCATCACATCGGACATA-3′	5′-GCTCCTCCCATAATACTCAGAACA-3′
COL-I ALP β-ACTIN	5′-CCAGAAGAACTGGTACATCAGCAA-3′ 5′-TAAGGACATCGCCTACCAGCTC-3′ 5′-TGGCACCCAGCACAATGAA-3′	5′-CGCCATACTCGAACTGGAATC-3′ 5′-TCTTCCAGGTGTCAACGAGGT-3′ 5′-CTAAGTCATAGTCCGCCTAGAGCA-3′
